# vB-ApyS-JF1, the First *Trueperella pyogenes* Phage, Shows Potential as an Alternative Treatment Strategy for *Trueperella pyogenes* Infections

This article has been retracted.

**DOI:** 10.3389/fmicb.2021.736304

**Published:** 2021-10-25

**Authors:** Yalu Ji, Liran Song, Zuoyong Zhou, Xiao Liu, Fengyang Li, Zhimin Guo, Yuan Guan, Li Yang, Xin Feng, Changjiang Sun, Liancheng Lei, Wenyu Han, Jingmin Gu

**Affiliations:** ^1^Key Laboratory of Zoonosis Research, Ministry of Education, College of Veterinary Medicine, Jilin University, Changchun, China; ^2^College of Veterinary Medicine, Southwest University, Chongqing, China; ^3^Department of Clinical Laboratory, The First Hospital of Jilin University, Changchun, China; ^4^Jiangsu Co-Innovation Center for the Prevention and Control of Important Animal Infectious Disease and Zoonose, Yangzhou University, Yangzhou, China

**Keywords:** phage therapy, *Trueperella pyogenes*, vB-ApyS-JF1, bacteremia, mice

## Abstract

Trueperella *pyogenes* (*T. pyogenes*) is an important opportunistic animal pathogen that causes huge economic losses to the animal husbandry industry. The emergence of bacterial resistance and the unsatisfactory effect of the vaccine have prompted investigators to explore alternative strategies for controlling *T. pyogenes* infection. Due to the ability of phages to kill multidrug-resistant bacteria, the use of phage therapy to combat multidrug-resistant bacterial infections has attracted attention. In this study, a *T. pyogenes* phage, vB-ApyS-JF1 (JF1), was isolated from sewage samples, and its whole genome and biological characteristics were elucidated. Moreover, the protective effect of phage JF1 on a mouse bacteremic model caused by *T. pyogenes* was studied. JF1 harbors a double-stranded DNA genome with a length of 90,130 bp (30.57% G + C). The genome of JF1 lacked bacterial virulence–, antibiotic resistance– and lysogenesis-related genes. Moreover, the genome sequence of JF1 exhibited low coverage (<6%) with all published phages in the NCBI database, and a phylogenetic analysis of the terminase large subunits and capsid indicated that JF1 was evolutionarily distinct from known phages. In addition, JF1 was stable over a wide range of pH values (3 to 11) and temperatures (4 to 50°C) and exhibited strong lytic activity against *T. pyogenes in vitro*. In murine experiments, a single intraperitoneal administration of JF1 30 min post-inoculation provided 100% protection for mice against *T. pyogenes* infection. Compared to the phosphate-buffered saline (PBS) treatment group, JF1 significantly (*P* < 0.01) reduced the bacterial load in the blood and tissues of infected mice. Meanwhile, treatment with phage JF1 relieved the pathological symptoms observed in each tissue. Furthermore, the levels of the inflammatory cytokines tumour necrosis factor-α (TNF-α), interferon-γ (IFN-γ), and interleukin-6 (IL-6) in the blood of infected mice were significantly (*P* < 0.01) decreased in the phage-treated group. Taken together, these results indicate that phage JF1 demonstrated great potential as an alternative therapeutic treatment against *T. pyogenes* infection.

## Introduction

*Trueperella pyogenes* (*T. pyogenes*), previously described as *Arcanobacterium pyogenes* or *Actinomyces pyogenes*, is an important opportunistic and prevalent pathogen worldwide (Zhang D. et al., 2017). *T. pyogenes* often causes purulent infections in pigs, cattle, sheep, and goats, primarily manifesting as pneumonia, arthritis, endocarditis, abortion, mastitis, subcutaneous abscess, and even animal death due to sepsis. Therefore, *T. pyogenes* conveys significant economic losses to the animal husbandry industry, primarily in cattle and swine breeding, causing a reduction in meat and milk yield, as well as decreased reproductive efficiency and sometimes the necessity to cull diseased animals (Rzewuska et al., 2019). In addition, as a zoonotic pathogen, *T. pyogenes* is also responsible for a number of human diseases, such as septicemia, endocarditis, arthritis, endemic leg ulcers, pneumonia, arthritis, various suppurative lesions, and abscesses (Rzewuska et al., 2019).

Antibiotics, such as beta-lactams, tetracyclines, and macrolides, have been used to treat liver abscesses caused by *T. pyogenes* (Jost and Billington, 2005; Zhang D. et al., 2017). However, antibiotic treatment of *T. pyogenes* infection is limited due to the emergence of resistant strains and the limited dosage of drugs in the infected site, such as abscesses (Rzewuska et al., 2019; Yang et al., 2020). Vaccines, such as inactivated recombinant vaccines (Hu et al., 2016; Zhang W. et al., 2017) and DNA vaccines (Huang et al., 2018), are another commonly used approach and have been thoroughly studied for use against *T. pyogenes* infection. However, there is only one commercial *T. pyogenes* vaccine available to date, and its immune protection is unsatisfactory based on a meeting report of the World Organization for Animal Health (OIE) *ad hoc* group, which discussed the prioritization of diseases and determined the vaccines that could reduce antimicrobial use in cattle, sheep, and goats (Yang et al., 2020). Hence, exploiting alternative efficient and safe strategies for controlling *T. pyogenes* infection is essential.

Bacteriophages (phages) are viruses that infect bacteria. The high specificity of phages against bacteria allows them to infect only host bacteria without damaging the commensal microbiota in the environment (Hyman and Abedon, 2010). Additionally, lytic phages are unable to persist *in vivo* and will be cleared automatically after the host bacteria are removed from the body (Loc-Carrillo and Abedon, 2011). Furthermore, the mechanism of action in phages is distinct from that of antibiotics, and phages have a bactericidal effect on multidrug-resistant bacteria, enabling their use to treat diseases caused by multidrug- resistant bacteria (Carlton, 1999). Based on these characteristics, phage therapy is regarded as an alternative therapeutic strategy to antibiotics for combating various bacterial infections in humans and animals (Cisek et al., 2017), such as pneumonia caused by *Streptococcus* pneumoniae (Qadir and Sajjad, 2017), bacteremia caused by *Enterococcus faecalis* and *Enterococcus faecium* (Cheng et al., 2017), burn wound infection caused by antibiotic-resistant pathogens (Kaur et al., 2019), and miscarriage caused by *Salmonella enterica serovar abortusequi* (Wang et al., 2020).

There is no known phage for *Trueperella*, aside from some bioinformatically predicted prophages (Machado and Bicalho, 2014). It has not stopped people from looking into phage therapy; for instance, Duarte et al. identified a T4 virus called vB_EcoM-UFV13 that could be used to disrupt *T. pyogenes* biofilms, although it was isolated from *E. coli* (da Silva Duarte et al., 2018). However, to our knowledge, phage therapy has not been used to treat infections caused by *T. pyogenes*.

In this study, vB-ApyS-JF1 (JF1), the first lytic *T. pyogenes* phage, was isolated using a *T. pyogenes* strain as the host. The genome and biological characteristics of this phage were assessed. Additionally, our treatment results using phage JF1 in a mouse bacteremia model provide a new strategy for the treatment of infections caused by *T. pyogenes*.

## Materials and Methods

### Ethics Statement

All animal experiments performed in this study strictly followed the National Guidelines for Experimental Animal Welfare (Ministry of Science and Technology of China 2006) and were approved by the Animal Welfare and Research Ethics Committee at Jilin University (Approved Number: SY202010031). All animals were treated humanely, and every effort was made to minimize suffering.

### Animals

Female BALB/C mice aged 6–8 weeks (18–20 g) were purchased from the Liaoning Provincial Laboratory Animal Resource Center, Shenyang, China. The mice were housed in a temperature-controlled animal room with a 12-h light/12-h dark cycle. Food and fresh water were available *ad libitum*.

### Bacterial Strains and Culture Conditions

All *T. pyogenes* strains used in this study are listed in Supplementary Table 1. All *T. pyogenes cells* were cultured in Martin broth medium with 10% fetal bovine serum under aerobic conditions and were identified by PCR-mediated amplification of a species-specific region of the 16S-23S rDNA intergenic spacer region (*ISR*) (GenBank: EU194563) (ISR-F: 5′-GTTTTGCTTGTGATCGTGGTGGTTATGA-3′, ISR-R: 5′-AA GCAGGCCCACGCGCAGG-3′) (Ulbegi-Mohyla et al., 2010) and by the available universal *sodA* gene–specific oligonucleotide (GenBank: AM949566) (sodA-F: 5′-CGAGCTCGCCGACGCTA TTGCT-3′, sodA-R 5′-GAGCATGAGAATCGGGTAAGTGC CA-3′) (Hijazin et al., 2011).

### Phage Isolation and Characteristics

Sewage samples were collected from the Changchun sewer system (Changchun, China). The *T. pyogenes* strain BS was used as a host to isolate phages from sewage samples. Briefly, 1 ml of strain BS was cultured with 100 ml sewage samples overnight in Martin broth medium with 10% fetal bovine serum at 37°C with shaking at 165 rpm. The culture was centrifuged at 9,000 × *g* for 10 min, and the supernatant was filtered through 0.22 μm pore size Millipore filters (Millipore, Bedford, MA, United States). The phage was detected using the spot assay (Chang et al., 2005) and was purified using the double-layer agar plate method (Ellis and Delbrück, 1939). Phage and host bacteria were added to 5 ml medium and co-cultured at 37°C for 16 h to amplify phages. The phage amplification solution was filtered through 0.22 μm filters, aliquoted into a 1.5 ml centrifuge tube, and stored at 4°C. The host spectrum of the phage was also determined using spot testing and the double-layer agar plate method using the *T. pyogenes* strains listed in Supplementary Table 1.

Phage JF1 was concentrated and purified as previously described with some modifications (Matsuzaki et al., 1992). Phage JF1 was amplified in 1,000 ml of Martin broth medium with 10% fetal bovine serum. Then, DNase I and RNase A were added to the mixture at a final concentration of 1 μg/ml and incubated on ice for 30 min. Next, NaCl was added to the mixture at a final concentration of 1 mol/L on ice for 1 h and then centrifuged at 10,000 × *g* for 20 min at 4°C. Polyethylene glycol 8,000 (final concentration of 0.1 g/ml) was added to the supernatant, incubated on ice for 8 h, and centrifuged at 10,000 × *g* for 20 min at 4°C. Phage JF1 was resuspended in 2 ml of SM buffer solution (pH 7.5, 50 mM Tris–HCl, 8 mM MgSO_4_, 0.1 M NaCl, and 0.01% (w/v) gelatin; Becton, Dickinson and Company, Franklin Lakes, NJ, United States). To purify phage JF1, the phage was mixed with an equal volume of chloroform and then centrifuged at 3,000 × *g* for 20 min at 4°C. The extraction was repeated three times.

The morphology of phage JF1 was observed according to a previous description (Xi et al., 2019). Briefly, the purified phage JF1 samples were dropped onto a grid surface, allowed to absorb for 15 min, and negatively strained with 2% phosphotungstic acid (PTA, 2% w/v). The morphology of phage JF1 was observed using an 80 kV transmission electron microscope (TEM) (JEOL JEM-1200EXII, Japan Electronics and Optics Laboratory, Tokyo, Japan).

A one-step growth curve of phage JF1 was determined as previously described with some modifications (Xi et al., 2019). Briefly, after mixing JF1 (100 μl, 1 × 10^8^ plaque forming unit (PFU)/ml) and *T. pyogenes* BS (1 ml, 1 × 10^8^ colony forming unit (CFU)/ml) at an MOI (multiplicity of infection: the ratio of phage number to host bacteria number) of 0.01, the mixture was incubated at 37°C for 5 min and then centrifuged at 10,000 × *g* for 5 min. The pellet was suspended in 10 ml of Martin broth medium and shaken at 165 rpm at 37°C. Samples were collected every 5 min for the first 30 min and then every 10 min until 60 min. Each sampling volume was 300 μl. Then, 150 μl samples were immediately passed through a 0.22 μm filter, and the titer was measured using the double-layer plate method after samples were diluted in sterile PBS (137 mM NaCl, 2.7 mM KCl, 50 mM Na_2_HPO_4_ and 10 mM KH_2_PO_4_, pH 7.4). Another 150 μl of sample was treated with 1% (*v/v*) chloroform for 30 min to release intracellular phages to determine the eclipse phase. All assays were performed in three independent experiments.

The pH sensitivity and thermal stability of phage JF1 were measured as previously described with some modifications (Chen et al., 2016). Briefly, phage JF1 (1 ml, 3 × 10^9^ PFU/ml) was mixed with SM buffer, which was adjusted to different pH values (pH = 1, 2, 3, 4, 5, 6, 7, 8, 9, 10, 11, 12), and incubated at 37°C for 1 h. Then, the samples were diluted in PBS, and the phage titers were determined using the double-layer plate method. Additionally, phage JF1 (1 ml, 3 × 10^9^ PFU/ml) was incubated at different temperatures (4, 25, 37, 40, 50, 60, and 70°C) for 120 min, and the samples were collected every 20 min. Phage titers were determined using the double-layer plate method. All assays were performed in three independent experiments.

### Genome Sequencing and Bioinformatics Analysis

The genome of phage JF1 was extracted using a viral genome extraction kit (Omega Bio-Tek Inc., Norcross, GA, United States). Whole-genome sequencing of JF1 was performed at the Beijing Genomics Institute using the 454 platform and assembled using Spades v. 3.6.2. Genomic termini and package mechanism were analyzed using PhageTerm (Garneau et al., 2017). Genes were initially predicted with the Rapid Annotation using Subsystem Technology (RAST) annotation server (Aziz et al., 2008). The genome of phage was analyzed using the phage AI tool. All of the predicted open reading frames (ORFs) were predicted and analyzed by BLASTp and GeneMarkS. The schematic diagrams of the gene functional module map were performed using CLC Main Workbench version 8.1 (CLC Bio-Qiagen, Aarhus, Denmark). The circle map of the phage genome was created using CGView^1^. The amino acid sequences of terminase large subunits and capsid proteins were aligned using BLASTp. The output was sorted according to the hit score, from which different phages with homology were selected, and their nucleic acid sequences were obtained. The sequences were then classified according to the NCBI taxonomy database. The gene sequences of the terminase large subunits and capsid proteins were aligned with reference gene sequences using the ClustalW program within the BioEdit 7.0.4.1 package. The maximum likelihood (ML) phylogenetic trees were constructed using their nucleic acid sequences with 1,000 bootstrap replicates.

### Mouse Model of Bacteremia

A mouse bacteremia model was established using previously described methods with minor modifications (Cheng et al., 2017). Briefly, to determine the minimal lethal dose (MLD) that causes mouse bacteremia and produces 100% mortality, 15 BALB/C mice were randomly divided into three groups (5 mice in each group) and intraperitoneally injected with different concentrations (3 × 10^7^, 3 × 10^8^, and 3 × 10^9^ CFU/mouse) of the *T. pyogenes* strain BS, respectively. The number of dead mice was recorded every day during the 7-day follow-up period. The MLD was determined, and 2 × MLD was the challenge dose.

To determine the rate of bacterial entry into the blood, three mice were randomly selected and intraperitoneally injected with 2 × MLD (6 × 10^8^ CFU/mouse) of *T. pyogenes* BS, and blood was collected from the tail vein of each mouse every 10 min for a total of 1 h after challenge. The blood was multiply diluted in sterile PBS, and colony counts were performed.

### Phage Therapy in a Murine Model of Bacteremia

To determine the protective effect of different titers of phage JF1 in the mouse bacteremia model, 60 mice were randomly divided into six groups containing 10 mice each. Mice in different groups were intraperitoneally injected with different titers (6 × 10^4^, 6 × 10^5^, 6 × 10^6^, or 6 × 10^7^ PFU/mouse) of phage JF1 in a single dose 30 min after the challenge, and mice in the control group were intraperitoneally injected with a sterile PBS buffer. In addition, 10 mice were intraperitoneally injected with 6 × 10^7^ PFU/mouse phage JF1 in a single dose at 1 h after the challenge. The number of dead mice was recorded every 12 h during the 7-day follow-up period.

One dose of phage (6 × 10^7^ PFU/mouse) was used to further evaluate the therapeutic effect on a mouse bacteremia model. In the experiment, all mice were randomly divided into four groups: phage treatment group A (mice were injected intraperitoneally with 6 × 10^8^ CFU/mouse *T. pyogenes* BS, and phage JF1 (6 × 10^7^ PFU/mouse) was administered after a 30-min challenge at a single dose), phage treatment group B (mice were injected intraperitoneally with 6 × 10^7^ PFU/mouse phage), PBS treatment group (mice were injected intraperitoneally with 6 × 10^8^ CFU/mouse *T. pyogenes* BS, and PBS was administered after a 30-min challenge), and normal group (mice with no treatment).

The bacterial loads and phage titers in the blood were subsequently determined. Briefly, three infected mice from phage treatment A and PBS treatment groups were euthanized with an injection of Fatal Plus (sodium pentobarbital, 100 mg/kg) 1, 2, 3, 4, 5, 6, 12, 18, 24, 30, 36, 42, 48, 60, 72, 84, and 96 h after challenge. Blood samples were collected from euthanized mice into 1.5 ml tubes containing 1 mM ethylene diamine tetraacetic acid (EDTA). Blood (100 μl) was taken for multiple dilutions to determine the bacterial load. In addition, the blood samples (300 μl) from the phage treatment groups were diluted multiple times, and the phage titer (including infected cells and free phages) was measured using the double-layer plate method. Moreover, three infected mice from phage treatment B were euthanized 5, 10, 15, 20, 25, and 30 min after injection. Blood samples (300 μl) were diluted multiple times, and the phage titer was measured using the double-layer plate method. Furthermore, *T. pyogenes* colonies were isolated from the blood of mice (3 mice) 48 h after infection in the phage treatment A group, and their sensitivity to phage was determined using the double-layer plate method.

The bacterial loads and phage titers in the lungs, livers, spleens, and kidneys were determined using another set of mice. Briefly, three mice from phage treatment or PBS treatment were euthanized 0.5, 6, 12, 18, 24, 48, 72, 96, and 120 h after challenge. The lung, liver, spleen, and kidney tissues from mice were weighed and suspended in filter-sterilized PBS. Then, each tissue was homogenized using sterile mortar pestles (JinTai, Changchun, China). Each homogenized suspension (100 μl) was serially diluted, and the colony counts were determined. In addition, each tissue grinding fluid sample (300 μl) from the phage treatment group was diluted multiple times, and the phage titer was measured using the double-layer plate method. Moreover, *T. pyogenes* colonies were isolated from each organ of mice (three mice) 48 h after infection in the phage treatment A group, and their sensitivity to phage was determined using the double-layer plate method.

A histopathological analysis of the lungs, livers, spleens, and kidneys of mice from the different treatment groups was performed. Briefly, three mice in each group were euthanized 12 h after challenge. The lungs, livers, spleens, and kidneys of the mice were removed and immediately placed in 4% formalin. The formalin-fixed tissues were subsequently stained with hematoxylin and eosin and analyzed by microscopy.

The levels of the cytokines tumour necrosis factor-α (TNF-α), interleukin-6 (IL-6), and interferon-γ (IFN-γ) in the blood from different groups were determined. Briefly, three mice in each group were euthanized 6, 12, 18, and 24 h after challenge. Blood samples were collected in 1.5 ml tubes and stored at 4°C overnight to separate the serum. The cytokine levels of TNF-α, IL-6, and IFN-γ in the serum were determined using enzyme-linked immunosorbent assay (ELISA) kits (BioLegend, San Diego, CA, United States).

### Statistical Analysis

SPSS version 13.0 software (SPSS, Inc., Chicago, IL, United States) was used for all statistical analyses. All experimental data were analyzed using one-way analysis of variance. Least—significant difference (LSD) (L), Student-Newman-Keuls (S-N-K) (S), and Tukey’s b (K) were used for *post hoc* tests. *P* < 0.05 was considered significantly different, and *P* < 0.01 was considered highly significantly different. Error bars represent the standard deviation (SD).

## Results

### Identification of the *T. pyogenes* Strain

The amplicon sizes of *ISR* and *sodA* were approximately 122 and 199 bp, respectively (Supplementary Figure 1), consistent with previous reports (Hijazin et al., 2011). BLAST analysis showed that the *ISR* and *sodA* gene sequences of the three strains were 100% identical to those of *T. pyogenes* strains that were identified in the GenBank database, such as CP050810.1 and CP033904.1, indicating that the isolated strains BS, S4, and Ty belong to *T. pyogenes.*

### Isolation, Characterization, and Host Range of Phage vB-ApyS-JF1

The purified phage JF1 produced a transparent plaque with a diameter of approximately 1–2 mm on an LB solid plate (Figure 1A). The TEM results showed that JF1 had an icosahedral head with a diameter of approximately 100 ± 3 nm (*n* = 3) and a non-contractile tail with a length of approximately 320 ± 3 nm (*n* = 3) (Figure 1B), indicating that it belongs to the *Siphoviridae* family. In addition, the one-step growth curve results revealed that the eclipse period of JF1 was approximately 5 min. The latent period was approximately 15 min, and the burst size was approximately 350 PFU/cell, indicating that JF1 had strong proliferation ability (Figure 1C). The results of the host profile measurement demonstrated that three of the six *T. pyogenes* strains tested were sensitive (Supplementary Table 1).

**FIGURE 1:** Characteristics of phage vB-ApyS-JF1 (JF1). **(A)** Plaques formed by JF1. **(B)** Phage JF1 was negatively stained with 2% phosphotungstic acid (PTA) and examined using transmission electron microscopy (TEM) at an accelerating voltage of 80 kV. The scale bar represents 100 nm. **(C)** One-step growth curve of JF1. The curve was determined when the multiplicity of infection (MOI) of JF1 was 0.01. The values represent the means and standard deviations (SDs) (*n* = 3).

### Stability of the Phage vB-ApyS-JF1

Phage JF1 titers remained unchanged after dissolution in SM buffer with a pH of 3∼11 for 1 h (Figure 2A). When the pH of SM buffer was less than 3 or greater than 11, the phage lost its lytic activity. In addition, JF1 maintained stability at 4–50°C. When the temperature reached 60°C, phage JF1 lost its activity completely after 1 h (Figure 2B). These results indicate that JF1 is stable over a wide range of pH values and temperatures.

**FIGURE 2:** Stability of phage JF1. **(A)** Stability of phage JF1 in different pHs. JF1 maintained stable activity after incubation in an SM buffer of pH 3–11 for 1 h. The values represent the means (*n* = 3) and the error bars the SD. **(B)** Stability of phage JF1 at different temperatures. JF1 maintained stable activity after incubation at 4–50°C for 1 h. The values represent the means and SD (*n* = 3).

### General Features of the Genome of Phage vB-ApyS-JF1

The coverage of the genome was 100% during genome assembly. The complete genome sequence of phage JF1 was deposited in GenBank and available in GenBank under accession number MW589261. Phage AI prediction analysis indicated that JF1 was a lytic phage. The analysis of genomic termini and packaging mechanism revealed that no termini could be detected for JF1, and no known packaging mechanism could be assigned to this phage (Supplementary Figure 2). The entire genome of phage JF1 was a 90,130 bp double-stranded DNA sequence with a G + C content of 30.57% (Supplementary Figure 3). The genome sequence of JF1 exhibited a low degree of coverage (<6%) with all other phages identified by BLASTp analysis. Two transfer-RNA-encoding genes were found in the genome (Supplementary Table 2). JF1 encoded 134 putative ORFs, with ATG (125/134), TTG (6/134), and GTG (3/134) serving as start codons. Among the 134 ORFs encoded by JF1, most of the phage JF1 genes were forward transcribed (1–2, 25–40, and 53–121 ORFs; the numbers represent the order of ORFs), while the rest were reverse transcribed (3–24, 41–52, and 122–134 ORFs). In addition, 89 genes encoded products that shared 31.53% ≦ identity ≦ 95.50% identity with known functional proteins, and the remaining 45 (33.58%) genes encoded products that did not match any published gene products in the NCBI database. Moreover, among all 89 predicted known functional proteins, 55 ORFs were homologous with previously identified bacteriophage genes, and 34 ORFs were homologs of proteins from bacteria (Supplementary Table 3).

According to the predicted functional proteins (Supplementary Table 3), a gene function module map of JF1 was drawn (Figure 3). The predicted functional proteins were divided into six modules according to their functions: nucleotide metabolism and replication, morphogenesis, host lysis, metabolic correlation, and unique and hypothetical proteins. The modules related to nucleotide metabolism and replication were composed of ORF13 (DNA packaging protein), ORF16 (assembly protease), ORF23 (HNH endonuclease), ORF63 (single-strand binding protein), ORF68 (DNA cytosine methyltransferase), ORF71–74 (ribonucleotide reductase alpha subunit, endonuclease, ribonucleotide reductase alpha subunit, ribonucleotide reductase beta subunit), ORF85 (DNA helicase), ORF87–89 (repair exonuclease, ribonuclease HI, LysR family transcriptional protein), ORF100 (nucleoside 2-deoxyribosyltransferase), and ORF106 (DNA polymerase). The modules related to metabolism contained ORF27 (serine/threonine protein phosphatase), ORF60 (response regulator), ORF62 (thioredoxin), ORF64 (ATP/GTP binding protein), ORF66 (tRNA methyltransferase), ORF94 (ATPase), ORF116 (guanylate kinase), ORF122 (tyrosine-type recombinase/integrase), ORF130 (peptidase G2), and ORF134 (tail tape measure protein).

**FIGURE 3:** Gene module map of JF1. Each arrow represents an open reading frame (ORF), and the direction of the arrow represents the direction of gene transcription. The predicted functional proteins were divided into six modules according to their functions. All modules are represented in different colors, and the putative functions and names of the genes are listed above.

The modules related to host lysis were composed of ORF123 (lysin) and ORF124 (holin). Moreover, 14 ORFs were found to encode proteins involved in morphogenesis, 2 of which were large terminase subunit proteins and a terminase small subunit protein encoded by ORF18, ORF19, and ORF22, respectively. In addition, ORF17 was predicted to encode a portal protein, and ORF134 was predicted to encode a tail tape measure protein. No drug resistance, pathogenicity, or lysogenic modules were found in the genome.

The terminase large subunit (ORF18 and ORF19) and capsid protein (ORF15) of phage JF1 were used to construct a phylogenetic tree. *Staphylococcus* phages were selected as the outgroup, and the ML was used to generate the phylogenetic tree. In Figure 4, the terminase large subunit (Figures 4A,B) and major capsid protein (Figure 4C) show that JF1 was evolutionarily distinct from other known phages, providing further support for the evolutionary divergence of JF1 from other phages (*Staphylococcus* phages PMBT8, VB-SauS-SA2, 6ec, vB_SepS_SEP9, *Lactobacillus* phages P1, Satyr, phiLdb, Ld3, ATCC 8014-B2, Ld17, P1174, Ld25A, Lenus, Nyseid, SA-C12, Ldl1, ViSo-2018a, ATCCB, and *Enterococcus* phages VFW, vipetofem, nattily, 9183) in terms of phylogeny, indicating that JF1 is a novel phage.

**FIGURE 4:** Phylogenetic trees were generated using the maximum likelihood (ML) method with 1,000 bootstrap replicates. **(A)** Phylogenetic tree based on the DNA of the terminase large subunits (ORF18) of JF1. **(B)** Phylogenetic tree based on the DNA of the terminase large subunits (ORF19) of JF1. **(C)** Phylogenetic tree based on the DNA of the capsid protein (ORF15) of JF1.

### Survival Outcomes of the Infected Mice

The bacterial load in the blood of the infected mice reached approximately 4.8 × 10^5^ CFU/ml 30 min after challenge and rose to 1.4 × 10^7^ CFU/ml (lethal dose) 1 h after challenge (Supplementary Figure 4). A single dose (3 × 10^8^ CFU/mouse) of *T. pyogenes* BS caused 100% mortality within 48 h, and the MLD of mice was determined to be 3 × 10^8^ CFU/mouse. When mice were challenged with a single dose of 2 × MLD (6 × 10^8^ CFU/mouse) of BS, as shown in Figure 5, all mice in the PBS treatment group died within 24 h after challenge. To determine the protective effect of phage JF1 on infected mice, a single dose of JF1 with different titers was intraperitoneally injected 30 min after the challenge. The results indicated that 6 × 10^4^ PFU/mouse phage JF1 had no protective effect on infected mice. When the phage titer was increased to 6 × 10^7^ PFU/mouse, phage JF1 provided 100% protection for infected mice (Figure 5). Therefore, the minimum therapeutic dose of phage JF1 was determined to be 6 × 10^7^ PFU/mouse. In addition, the protection rate of a single dose of 6 × 10^7^ PFU/mouse of JF1 on infected mice 1 h after the challenge was 20% (Supplementary Figure 5).

**FIGURE 5:** Survival rates of infected mice. Mice were intraperitoneally challenged with *T. pyogenes* BS (6 × 10^8^ CFU/mouse), and infected mice were intraperitoneally treated with different doses of JF1 30 min postinfection. The control group was treated with the same amount of sterile PBS. Compared to the other groups, 6 × 10^7^ PFU/mouse JF1 significantly improved the survival rate of infected mice. Each group contains 10 mice. **P < 0.01.

### vB-ApyS-JF1 Reduced the Bacterial Load in the Mouse Bacteremia Model

The bacterial load in the blood of the mice in the PBS treatment group reached approximately 1.5 × 10^7^ CFU/mL 1 h after the challenge. As time passed until the mice died, the bacterial load in the blood of the mice stabilized at approximately 2 × 10^7^ CFU/ml. Compared to the PBS treatment group, the bacterial load in the blood of mice was reduced by approximately 2 log in the JF1 treatment group after 1 h of infection. The bacterial load in the JF1 treatment group was gradually eliminated 48 h after the challenge (Figure 6A). In addition, the phage titer in the blood of mice rose briefly and then gradually decreased with the reduction in the number of bacteria and was finally almost entirely eliminated 96 h postinfection (Figre 6B). The same dose of phage JF1 (6 × 10^7^ PFU/mouse) was injected intraperitoneally into uninfected mice. The effective phage titers in the blood of the mice plummeted (1 log −2 log) after 5 min, and no phage was detected after 30 min (Supplementary Figure 6). Furthermore, a total of 15 *T. pyogenes* colonies were isolated from the blood of three mice infected for 48 h in the phage treatment group, and the results showed that they maintained their sensitivity to phage JF1 (data not shown).

**FIGURE 6:** Determination of bacterial load and phage titers in blood samples of mice. Blood samples were collected from mice of each group 1, 2, 3, 4, 5, 6, 12, 18, 24, 30, 36, 42, 48, 60, 72, 84, and 96 h after challenge. Three mice from each group were euthanized at each time point. **(A)** Each blood sample was diluted multiple times, and the colony counts were determined. **(B)** The titers of phage JF1 were measured using the double-layer plate method. The values represent the means and SDs (*n* = 3). **P < 0.01.

The bacterial load in the lung, liver, spleen, and kidney tissues of mice in the PBS treatment group reached approximately 7.2 × 10^6^ CFU/mg (lung) (Figure 7A), 1.3 × 10^6^ CFU/mg (liver) (Figure 7B), 2.8 × 10^5^ CFU/mg (spleen) (Figure 7C), and 8.1 × 10^4^ CFU/mg (kidney) (Figure 7D) 6 h postinfection. Compared to that, the bacterial load in each tissue was significantly (*P* < 0.01) reduced in response to JF1 treatment, being approximately 4.9 × 10^2^ CFU/mg (lung) (Figure 7A), 2.5 × 10^2^ CFU/mg (liver) (Figure 7B), 5.6 × 10^4^ CFU/mg (spleen) (Figure 7C), and 2.1 × 10^2^ CFU/mg (kidney) (Figure 7D). When the mice had been infected for 18 h, the bacterial load of the lung, liver, spleen, and kidney tissues of the mice in the PBS treatment group reached approximately 3.4 × 10^5^ CFU/mg (lung) (Figure 7A), 5.9 × 10^5^ CFU/mg (liver) (Figure 7B), 2.3 × 10^5^ CFU/mg (spleen) (Figure 7C), and 7.2 × 10^4^ CFU/mg (kidney) (Figure 7D). However, the bacterial load in each tissue was significantly (*P* < 0.01) reduced in response to JF1 treatment, being approximately 8.1 × 10^1^ CFU/mg (lung) (Figure 7A), 5.8 × 10^1^ CFU/mg (liver) (Figure 7B), 1.1 × 10^1^ CFU/mg (spleen) (Figure 7C), and 3.1 × 10^1^ CFU/mg (kidney) (Figure 7D). The bacterial load in each tissue of the infected mice was gradually cleared by 96 h after JF1 treatment (Figures 7A–D). In addition, phage titers in the tissues of mice in the phage treatment group decreased gradually following the decrease in bacterial load. Phage JF1 in kidney tissue was cleared approximately 50 h after treatment (Figure 7H), JF1 in lung and liver tissue was cleared approximately 96 h after treatment, and JF1 in the spleen was cleared approximately 120 h after treatment (Figures 7E–G). Moreover, a total of 21 *T. pyogenes* colonies were isolated from the organs of three mice infected for 48 h in the phage treatment group, and the results showed that they were sensitive to phage JF1 (data not shown).

**FIGURE 7:** Bacterial load and phage titers in mouse organs. The lung, liver, spleen, and kidney pieces of mice from each group were harvested and homogenized 0.5, 6, 12, 18, 24, 48, 72, 96, and 120 h after challenge. A total of 36 mice were used in this experiment. Three mice from each group were euthanized at each time point. **(A–D)** Fluid from each ground tissue was diluted multiple times, and the colony counts were determined. **(E–H)** The titers of phage JF1 were measured using the double-layer plate method. The values represent the means and standard deviations (SDs) (*n* = 3). *P < 0.05; **P < 0.01.

### vB-ApyS-JF1 Alleviates Injury and Inflammation in a Mouse Bacteremia Model

According to the histopathological observations, compared to normal mouse tissues, the lungs and spleen of mice in the PBS treatment group were more severely injured, with apparent neutrophil infiltration in the lungs, hemorrhage in the lung interstitium, and severe congestion. Some lymphocytes in the spleen tissue were lost, some cells were disintegrated and fragmented, a few cells were necrotic, and red blood cells were increased. The kidneys and liver sinusoids exhibited a small amount of bleeding. However, the phage treatment group exhibited significantly alleviated pathological damage in each tissue, and the organization scoring criteria used have been previously described (Wu et al., 2017). There was no neutrophil infiltration in the lung tissue, and no bleeding was observed in the lung interstitium. The lymphocytes in the spleen tissue were intact, and red blood cells were almost invisible. In addition, there was almost no congestion in the kidneys or liver sinuses. These results were all similar to those observed in normal tissues (Figure 8). In addition, the levels of the inflammatory cytokines TNF-α, IL-6, and IFN-γ in the blood were measured. As shown in Figure 9, the levels of TNF-α, IL-6 and IFN-γ were increased in the blood of infected mice 18 h postinfection compared to those of healthy mice, reaching approximately 1.8 × 10^3^ pg/ml, 7.9 × 10^3^ pg/ml, and 1.9 × 10^4^ pg/ml, respectively. However, compared to those in the PBS treatment group, the levels of these cytokines in the JF1 treatment group were reduced by approximately 3 log (TNF-α), 1 log (IL-6), and 3 log (IFN-γ) and were similar to those in the control group (Figure 9).

**FIGURE 8:** Histopathology of different tissues. The lungs, livers, spleens, and kidneys of mice from each group were removed 12 h after challenge and immediately placed in 4% formalin. The formalin-fixed tissues were then processed, stained with hematoxylin and eosin, and analyzed by microscopy. The main lesions of each tissue were indicated by arrows.

**FIGURE 9:** Levels of TNF-α, IL-6, and IFN-γ in the blood of mice. All mice were from three groups: phage (vB-ApyS-JF1) treatment group (mice were injected with *T. pyogenes* BS, and phage JF1 was administered 30 min after challenge in a single dose); PBS treatment group (mice were injected intraperitoneally with *T. pyogenes* BS, and PBS was administered 30 min after challenge). The normal group without any treatment was used as a control. Three mice from each group were euthanized at each time point. Blood samples were collected from mice of each group 6, 12, 18, and 24 h after challenge. The levels of TNF-α **(A)**, IL-6 **(B)**, and IFN-γ **(C)** cytokines in the blood were measured. Blood samples from healthy mice were used as controls (normal group). The values represent the means and SDs (*n* = 3). **P < 0.01.

## Discussion

To date, phages have long shown promise as potential antibacterial therapies, but to the best of our knowledge, there have been no reports on phages of *T. pyogenes*. In this study, we used *T. pyogenes* BS as the host bacteria to isolate the first *T. pyogenes* phage, JF1. The entire genome of phage JF1 was analyzed, its general biology was characterized, and the therapeutic effect of the phage on a mouse bacteremia model was evaluated.

When comparing the whole genome of phage JF1 in the NCBI database, we found that the genome had only 6% coverage with published phages, indicating that the JF1 genome is largely unique compared to published phage genomes. Moreover, among all ORFs, 45 (33.58%) gene-encoding products did not match any published gene products in the NCBI database, confirming the novelty of phage JF1 and supplementing the genome information of phages in the NCBI Genome database. Meanwhile, the functional properties of these unknown proteins and their role in phage survival and replication are unclear and need to be further studied. Among all the predicted proteins that matched published gene products, we did not find any related to virulence-, antibiotic resistance-, or lysogenesis-related genes, which is conducive to the use of the phage in therapeutic research.

One putative lysin gene (ORF 123) in the JF1 genome has 67.46% amino acid identity with *Staphylococcal* phage vB_SauS_IMEP5 (GenBank accession KX156762.1). Among all predicted proteins of JF1, only the lysin gene exhibited homology with phage vB_SauS_IMEP5. However, according to the phylogenetic tree analysis of the JF1 large subunit terminase, no correlations were found between vB_SauS_IMEP5 and JF1, which may be due to the modularity of phages. Most phages with tails use two essential proteins (lysin and holin) to achieve lysis (Wang et al., 2000). The holin protein is adjacent to lysin in the genome of JF1. Therefore, JF1 may also use a holin–endolysin strategy to lyse the host cell to liberate progeny virions. Many studies have indicated that lysin has many advantages over phages and conventional antibiotics and has become a new strategy to control food safety, environmental purification, and bacterial infection (Nelson et al., 2012). Therefore, it is necessary to conduct further research on the phage lysin of *T. pyogenes*. Among all ORFs, five proteins were annotated as tail proteins. Of all the structural proteins in the phage, the tail structure is a key factor in host specificity and infection process (Nobrega et al., 2018; Yehl et al., 2019). Differences in the tail proteins of phages may result in different host profiles and lytic activities (Yehl et al., 2019). Whether these five tail proteins of phage JF1 play a key role in phage lysis activity and host spectrum needs further study. In this study, only six *T. pyogenes* strains were used to test the host profile, and half of the *T. pyogenes* strains could be infected by phage JF1, including the standard strain ATCC49698. However, a larger number of strains are needed to further determine the host spectrum of JF1.

In *in vitro* experiments, the short latent period and high burst size of JF1 indicated its high propagation and lysis efficiency. The stability of phages under various conditions is a key factor in evaluating their application potential (Sharma et al., 2017). JF1 was stable over a wide pH values (pH 3–11) and temperature range (4–50°C), which is beneficial to the phage for maintaining its activity in different environments. Antibodies and phages have been considered for use as bioprobes to detect bacteria (Sorokulova et al., 2005). Compared to antibodies, phages possess some significant benefits in that phages are more resistant to higher temperature and/or pH fluctuations (Anany et al., 2011). Therefore, phage JF1 may be useful as a biological probe to detect *T. pyogenes*. In addition, the strong acid resistance of phage JF1 was conducive to its resistance to the gastric acid environment and has been used as a treatment of gastrointestinal diseases (Xue et al., 2020). All of these biological characteristics of JF1 indicate its great potential against *T. pyogenes*.

In the *in vivo* experiments, a single dose of 6 × 10^7^ PFU/mouse JF1 provided 100% protection to infected mice 30 min after challenge. Generally, different treatment times after infection have different effects. In fact, the protection rate of a single dose of 6 × 10^7^ PFU/mouse of JF1 on infected mice 1 h after the challenge was also measured, and the protection rate was only 20% (Supplementary Figure 4). These results are similar to the results of Zhang et al., who found that administering phages IME-EF1 (the latent period was 25 min) 30 min post-inoculation of *Enterococcus faecalis* led to therapeutic efficacy with a survival rate of 60%, whereas administering phages at 4 h provided 40% protection rate (Zhang et al., 2013).

The results of the bactericidal activity of phage JF1 *in vitro* and *in vivo* revealed that it was efficient and rapid, which is conducive to the elimination of pathogenic bacteria by phages. However, the pharmacological results of therapeutic drugs usually depend on the concentration of the drug and/or its active metabolites in the body. Physiologically based pharmacokinetics are a quantitative tool for understanding the concentration of drugs in the body (Ishimoto and Kato, 2016). Since phages replicate in the body, the pharmacokinetics of phages are essentially different from those of chemical drugs in the presence of sensitive bacteria (Abedon, 2014). In this study, the titers of phage JF1 in the blood of infected mice reached approximately 10^8^ PFU/ml 30 min after treatment, which was higher than the therapeutic dose administered (6 × 10^7^ PFU/mouse). This may be related to the growth characteristics of the phage. The one-step growth curve study of phages *in vitro* shows that the phage completes a lysis cycle within 30 min. If phage JF1 works as quickly *in vivo* as *in vitro*, the phage can proliferate rapidly within only 30 min. In addition, as the bacterial counts decrease and the bacteria are eventually eliminated, the titers of JF1 phage in the blood and organ tissues of the infected mice are also reduced. Phages rely on the host to replicate. When the number of host bacteria in the environment decreases, the amount of phage decreases (Diaz-Munoz and Koskella, 2014). Moreover, with the participation of the innate immune system and the complement system, phages are eventually eliminated (Dabrowska, 2019). When there were no phage-sensitive bacteria in healthy mice, after the same dose of phage was injected intraperitoneally, the phage titer in the blood of the mice was plummeted and was quickly cleared within half an hour (Supplementary Figure 5). This result is similar to previous research and suggests a very rapid mechanism of capturing or neutralizing the phages (Sulkin et al., 1957; Bartell et al., 1965; Inchley, 1969). In fact, we also measured the sensitivity of bacteria in the infected mice at the later stage of treatment in response to phage, and we did not observe the emergence of resistant bacteria. These are exciting findings, and we will perform additional experiments in future research.

In summary, *T. pyogenes* phage JF1 exhibits strong lytic activity and stability *in vitro* and exerted strong therapeutic effects against bacteremia caused by *T. pyogenes* infection. More research is needed to evaluate the potential of phage JF1 against *T. pyogenes* infection. Studies have shown that *T. pyogenes* can form biofilms and develop resistance to sensitive antibiotics (Olson et al., 2002; Zhao et al., 2013). *Escherichia* phage vB_EcoM-UFV13 was shown to prevent biofilm formation by *T. pyogenes* but was not able to infect or lyse *T. pyogenes* (da Silva Duarte et al., 2018). Whether phage JF1 can prevent and eliminate *T. pyogenes* biofilms is worthy of further study.

## Conclusion

In this study, *T. pyogenes* phage vB-ApyS-JF1 was characterized, and the therapeutic effect of phage JF1 on a mouse bacteremia model was investigated. Genome and phylogenetic tree analyses demonstrated that JF1 is a novel phage. *In vitro* studies indicated that JF1 exerts strong lytic activity and exhibited high stability in terms of temperature and pH. *In vivo* studies demonstrated that a single dose of JF1 had 100% protection against bacteremia in mice. A single dose of phage JF1 significantly reduced the bacterial load in the blood and primary organs of the infected mice in a short time and alleviated pathological damage to the tissues. The titer of JF1 in the blood and tissues was eliminated along with the removal of bacteria. In addition, JF1 reduced the levels of inflammatory factors in the blood. Therefore, phage JF1 shows great potential for controlling *T. pyogenes* infection.

## Data Availability Statement

The datasets presented in this study can be found in online repositories. The names of the repository/repositories and accession number(s) can be found in the article/Supplementary Material.

## Ethics Statement

The animal study was reviewed and approved by the Animal Welfare and Research Ethics Committee at Jilin University.

## Author Contributions

ZZ, XL, FL, ZG, YG, and LY assisted in carrying out the experiment. YJ and LS wrote the manuscript. XF, CS, LL, WH, and JG helped with the design of experimental ideas and the revision of manuscripts. All authors contributed to the article and approved the submitted version.

## Conflict of Interest

The authors declare that the research was conducted in the absence of any commercial or financial relationships that could be construed as a potential conflict of interest.

## Publisher’s Note

All claims expressed in this article are solely those of the authors and do not necessarily represent those of their affiliated organizations, or those of the publisher, the editors and the reviewers. Any product that may be evaluated in this article, or claim that may be made by its manufacturer, is not guaranteed or endorsed by the publisher.

## Footnotes

1
http://wishart.biology.ualberta.ca/cgview/
